# Risk Factors of Urinary Tract Infection in Pediatric Patients with Ureteropelvic Junction Obstruction after Primary Unilateral Pyeloplasty

**DOI:** 10.1155/2022/3482450

**Published:** 2022-07-15

**Authors:** Hongyang Wang, Chunsheng Hao, Dongsheng Bai

**Affiliations:** Department of Urology, Children's Hospital, Capital Institute of Pediatrics, Beijing, China

## Abstract

**Objective:**

Ureteropelvic junction obstruction (UPJO) represents to a leading cause of fetal hydronephrosis, which is associated with urinary tract infection (UTI) and urinary stone disease. This study is aimed at investigating risk factors of UTI in pediatric patients with UPJO after primary unilateral pyeloplasty.

**Methods:**

The records of a consecutive series of patients undergoing primary pyeloplasty at a single institution between June 2015 and November 2021 were retrospectively reviewed. Demographic and clinical characteristics, including age, gender, weight, height, body mass index (BMI), creatinine (Cr), blood urea nitrogen (BUN), estimated glomerular filtration rate (eGFR), neutrophil ratio, lymphocyte ratio, neutrophil/lymphocyte ratio, renal pelvis anteroposterior diameter (APD), renal cortex thickness, caliectasis, open or laparoscopic pyeloplasty, and internal drainage or external drainage, were collected and analyzed. The incidence of postoperative UTI and its risk factors was analyzed.

**Results:**

A total of 504 patients were enrolled in the study, and they were classified into the UTI group (*n* = 188) and non-UTI group (*n* = 361). Univariate analysis of the incidence of UTI revealed that age, gender, weight, height, BMI, surgical modality, Cr level, BUN level, neutrophil ratio, lymphocyte ratio and neutrophil/lymphocyte ratio, renal cortex thickness, and postoperative drainage modality were associated with UTI incidence after pyeloplasty in pediatric patients with UPJO. Multivariate analysis revealed that male gender, <19 months, weight < 11.5 (kg), height < 83 (cm), BMI < 17.09, BUN > 4.08 (mmol/L), and internal drainage were risk factors of postoperative UTI in pediatric patients with UPJO.

**Conclusion:**

Our study demonstrated that male gender, <19 months, weight < 11.5 (kg), height < 83 (cm), BMI < 17.09, BUN > 4.08 (mmol/L), and internal drainage were risk factors of UTI in pediatric patients with UPJO after primary unilateral pyeloplasty, which may provide reference for prophylactic antibiotics for those patients with risk factors.

## 1. Introduction

With the widespread use of obstetric ultrasonography, antenatal hydronephrosis has been reported more frequently, accounting for 1-4% of all pregnancies [1]. Antenatal hydronephrosis is usually asymptomatic, and one third of the patients become an important clinical issue [2]. The etiology of antenatal hydronephrosis involves ureteropelvic junction obstruction (UPJO), transient or physiologic hydronephrosis, and vesicoureteral reflux [3]. UPJO is a medical disorder arising from partial or complete obstruction of urine transport, increasingly being the most common cause of hydronephrosis in pediatric populations [4]. In the last decades, we have witnessed significant advancements on surgical techniques for the treatment and management of UPJO, from open approaches, laparoscopic techniques, to final robot-assisted approaches in 2002 [5, 6]. Open pyeloplasty is still the common surgical approach for UPJO, with a success rate of 90%, which involves a large flank incision and leads to prolonged postoperative recovery [7]. Of note, laparoscopic techniques, either by transperitoneal or retroperitoneal approaches with or without robotic assistance, have rapidly gained favors in urology practice [8]. At present, all these approaches are clinically used for surgical management of UPJO, and minimal invasive treatment options, laparoscopic and robot-assisted pyeloplasty, are often claimed to outperform open pyeloplasty in terms of early recovery and lower complication rates, whereas open pyeloplasty exhibits a shorter operation time [9]. However, anterograde and retrograde endopyelotomies showed inferior outcomes, except risk of bleeding, compared with laparoscopic techniques [10].

There were three common postoperative complications following pyeloplasty, including urinary tract infection (UTI), prolonged urinary leak, and wound infection. The incidence of UTI is up to 7.8%-10.0% when stents are left [11, 12]. Accordingly, prescription of prophylactic oral antibiotics is suggested by some pediatric urologists to decrease the risk of UTI following pyeloplasty during the placement of double-J stents [13]; although, very few patients with ureteral stents, particularly those with stent duration lasting no more than 3 months, show clinically symptomatic UTI [14]. Whether there are other risk factors of UTI in pediatric patients with UPJO after primary unilateral pyeloplasty is largely unknown. Therefore, it is necessary to investigate risk factors of UTI in pediatric patients with UPJO after primary unilateral pyeloplasty, so as to direct prevention of postoperative UTI.

## 2. Materials and Methods

### 2.1. Patient Selection

We retrospectively reviewed data of a consecutive series of pediatric patients who had undergone primary unilateral pyeloplasty at the Capital Institute of Pediatrics between June 2015 and November 2021, and the protocol was conducted with the human subjects understanding and consent, as well as approved by the Institutional Review Board. Exclusion criteria were as follows: those aged >18 years at their surgeries, bilateral repair or solitary kidney, taking antibiotics at the time of surgery, positive preoperative urinalysis and urine culture, and failure of surgery. The diagnosis of UPJO was determined according to ultrasonography, magnetic resonance urography (MRU), computed tomography urography (CTU), or radionuclide imaging. Among 504 pediatric patients, 188 cases were diagnosed with UTI by urinalysis and urine culture according to the European Association of Urology (EAU) guidelines on Pediatric Urology published in 2015 in European Urology [15].

### 2.2. Indications for Surgery

Indications for surgery included an obstructive drainage pattern with a T1/2 > 20 min on diuretic renal scan concomitant with reduced relative renal function < 40% in the affected kidney, increasing hydronephrosis on serial ultrasounds, and/or a decline in relative renal function more than 10% on serial renal scans.

### 2.3. Surgical Technique and Postoperative Care

Open pyeloplasty was approached extraperitoneally through a posterior incision. The muscle layers were split to identify the Gerota fascia. Following fascia incision, the renal pelvis was exposed. Repair was performed with absorbable 6-0 or 7-0 polyglactin sutures. Double-J stents were placed in an antegrade fashion through the cystoscopy. A perinephric drain was left in place until the drainage is <10 ml within 24 h. Urethral catheter was left indwelling until discharge.

Laparoscopic pyeloplasty was performed with the transperitoneal approach by laparoscopic surgeons who have the same skills and experiences with regard to pyeloplasty surgery. At the beginning of the procedure, cystoscopy and retrograde pyelogram with stent placement were carried out. The operations were conducted through 3 ports with two working ports (3 or 5 mm) and a 5 mm port for the camera. The renal pelvis was exposed and then drawn out of the abdominal cavity through the slightly extended camera port site. Repair was subsequently made with 5-0 or 6-0 absorbable polyglactin sutures or 6-0 polydioxanone. Double-J stents, perinephric drain, and urethral catheter were left and removed just like in open pyeloplasty.

### 2.4. Data Collection

Demographic and clinical characteristics, including age, gender, weight, height, body mass index (BMI), creatinine (Cr), blood urea nitrogen (BUN), estimated glomerular filtration rate (eGFR), neutrophil ratio, lymphocyte ratio, neutrophil/lymphocyte ratio, renal pelvis anteroposterior diameter (APD), renal cortex thickness, caliectasis, open or laparoscopic pyeloplasty, and postoperative drainage (internal drainage or external drainage), were collected and analyzed.

### 2.5. Statistical Analysis

Categorical data were shown as frequencies or percentage and compared using chi-square test. Continuous data were examined by Shapiro Wilk test for normal distribution. Nonparametric continuous data were shown as median (quartile 25%, quartile 75%) and analyzed by Mann–Whitney *U* test. Logistic regression analysis was performed to evaluate risk factors of UTI after pyeloplasty. Statistical analysis was performed using SPSS software package (version 21) (IBM Corp., Armonk, NY, USA), and *P* < 0.05 was considered statistically significant.

## 3. Results

### 3.1. Demographic and Clinical Characteristics of Patients

A total of 504 pediatric patients undergoing pyeloplasty due to UPJO were included in this study. They were aged 19.00 (5.35, 60.00) months. Among them, there were 407 males (80.75%) and 97 females (19.25%). 223 cases (44.25%) underwent laparoscopic pyeloplasty, among which 96 (41.56%) developed UTI, and 281 cases (55.75%) received open pyeloplasty, among which 92 (33.09%) developed UTI. 96 cases (19.05%) showed caliectasis, 355 cases (70.44%) received internal drainage, and 149 cases (29.56%) received external drainage. Postoperative UTI was found in 188 pediatric patients (37.30%). Other demographic and clinical characteristics of patients are listed in Table 1.

### 3.2. Univariate Analysis of the Incidence of UTI

Demographic and clinical characteristics of patients grouped by UTI and non-UTI are listed in Table 2. It was found that pediatric patients with postoperative UTI were younger than those without (*P* < 0.001). A higher proportion of male pediatric patients was found to suffer from postoperative UTI (*P* = 0.017). The pediatric patients with postoperative UTI exhibited decreased weight and height compared to those without (*P* < 0.001), and significant difference was also found in BMI (*P* = 0.007). More pediatric patients receiving laparoscopic pyeloplasty seem to suffer postoperative UTI than those receiving open pyeloplasty (*P* = 0.018). There were remarkable differences in terms of Cr level, BUN level, neutrophil ratio, lymphocyte ratio, and neutrophil/lymphocyte ratio between pediatric patients with postoperative UTI and those without (*P* < 0.001). The renal cortex was thinner in pediatric patients with postoperative UTI than those without (*P* < 0.001). More pediatric patients receiving internal drainage seem to suffer from postoperative UTI than those receiving external drainage (*P* < 0.001). No significant difference was found in eGFR, APD, and caliectasis between pediatric patients with postoperative UTI and those without (*P* > 0.05). Univariate analysis of the incidence of UTI revealed that age, gender distribution, weight, height, BMI, surgical modality, Cr level, BUN level, neutrophil ratio, lymphocyte ratio and neutrophil/lymphocyte ratio, renal cortex thickness, and postoperative drainage modality were related to the incidence of UTI after surgery in pediatric patients with UPJO.

### 3.3. Risk Factors of Postoperative UTI in Pediatric UPJO Patients

We performed multivariate analysis on the incidence of postoperative UTI in pediatric UPJO patients, and age (assigned as actual values), gender (assigned as 1 = male; 2 = female), weight (assigned as actual values), height (assigned as actual values), BMI (assigned as actual values), surgical modality (assigned as 1 = open pyeloplasty; 2 = laparoscopic pyeloplasty), Cr level (assigned as actual values), BUN level (assigned as actual values), neutrophil ratio (assigned as actual values), lymphocyte ratio (assigned as actual values) and neutrophil/lymphocyte ratio (assigned as actual values), renal cortex thickness (assigned as actual values), and postoperative drainage modality (assigned as 1 = internal drainage; 2 = external drainage) were included. It was revealed that male gender, <19 months, weight < 11.5 (kg), height < 83 (cm), BMI < 17.09, BUN > 4.08 (mmol/L), and internal drainage were found as risk factors of postoperative UTI in pediatric UPJO patients (Table 3).

## 4. Discussion

In the past decade, we have witnessed an increasing application of minimally invasive pyeloplasties from 0.34 to 11.7% [16, 17]. However, open pyeloplasty is still the most common operation for UPJO in pediatric urology, and laparoscopic surgery seems to be available in high-class pediatric hospitals. In this study, we analyzed a large case series who underwent primary pyeloplasty to identify risk factors of postoperative UTI in children. Among them, 188 children were found to have UTI, accounting for 37.30%, which was much higher than 7.8%-10% in the previous reports [11, 12], probably due to the exclusion of pediatric patients who took antibiotics at the time of surgery in our study. As shown by our data, although more pediatric patients receiving laparoscopic pyeloplasty seem to suffer postoperative UTI than those receiving open pyeloplasty, we failed to prove that laparoscopic pyeloplasty would increase the risk of postoperative UTI.

In our study, multivariate analysis revealed that male gender, <19 months, weight < 11.5 (kg), height < 83 (cm), BMI < 17.09, BUN > 4.08 (mmol/L), and internal drainage were risk factors of postoperative UTI in pediatric UPJO patients, suggesting that younger boys with lower weight or height, lower BMI, higher BUN, or internal drainage may require more attention regarding postoperative UTI. A previous study demonstrated that uropathogens isolated from male urolithiasis patients were more resistant to antimicrobials than female, revealing the presence of sex differences with regard to microbial spectrum and antibiotic sensitivity [18]. Consistent with our study, gender difference was also observed in patients with UTI after retrograde upper urinary lithotripsy [19]. More similarly, Wang et al. found that infants and young children with double-J catheter retention exhibited a higher risk of UTI, largely due to Gram-negative bacilli, and male sex was also a risk factor of UTI [20]. In addition to gender difference, younger age was also considered as a risk factor of UTI, consistent with the previous finding [21]. Badawy et al. reported that given the limited space for manipulation, children aged <3 months are supposed to receive open pyeloplasty, and children aged <2 years are more suitable for retroperitonoscopic pyeloplasty [22].

As shown by our study, lower weight, height, and BMI were associated with the incidence of UTI following either open or laparoscopic pyeloplasty. It was once reported that children with lower weight (<10 kg) and intraoperative complications with nephrostomy tubes were risk factors of higher Clavien grade postoperative complications [11]. Also, for children ≤ 10 kg, laparoscopic pyeloplasty confers a high successful rate concomitant with a low rate of complications [23]. In Kose et al.'s study, they included 178 (134 males, 44 females) patients and found postnatal early circumcision of infants with antenatal hydronephrosis which appears to reduce the risk of UTI and nutritional disturbances enabling normal growth [24]. Deterioration in height began early in the course of disease and was worsening with the decline of renal function [25]. Malaki and his team reported a significant association between growth quality (weight height index) and UTI [26]. However, to our knowledge, we first demonstrated that BMI < 17.09 was a risk factor of UTI after primary unilateral pyeloplasty.

The serum level of BUN is commonly used for estimation of renal function, and impaired renal function has been found to be related to UTI [27], similar to our finding. Of note, internal drainage after pyeloplasty was demonstrated to be a risk factor of postoperative UTI in our study. Previous evidence showed that the risk of febrile UTI could be lowered if the duration of ureteral stent placement was less than 21 days, and operation time was less than 75 min in patients with obstructive pyelonephritis [28]. It is believed that duration of ureteral stent retention significantly increases the risk of UTI. In the study of Klis et al., they noted a remarkable correlation between the duration of ureteral stent placement and urine culture, and double-J catheter retention was related to an increased risk of bacterial colonization [29].

In our study, the association of neutrophil/lymphocyte ratio and renal cortex thickness with UTI after primary unilateral pyeloplasty was innovatively investigated. Univariate analysis showed that neutrophil/lymphocyte ratio and renal cortex thickness were associated with UTI after primary unilateral pyeloplasty. However, multivariate analysis failed to support neutrophil/lymphocyte ratio and renal cortex thickness as independent risk factors of UTI after primary unilateral pyeloplasty. Due to retrospective nature of the study and the inevitable bias, this finding remains to be further verified by more well-designed studies.

Limitation should be noted when interpreting this study. First, due to pediatric patient admission in the 6-year period, included pyeloplasties were done by several surgeons. Although they all had similar experience with open or laparoscopic pyeloplasty surgery, bias on surgical outcomes may be considered. Second, the exact time of the complications was unable to be recorded in half of the patients during the follow-up, and the follow-up time was limited. Third, our study was retrospective in nature, and we failed to confirm compliance for the full duration of ureteral stenting. Our findings remain to be further verified by well-designed prospective studies with longer follow-up.

## 5. Conclusion

In summary, male gender, <19 months, weight < 11.5 (kg), height < 83 (cm), BMI < 17.09, BUN > 4.08 (mmol/L), and internal drainage were risk factors of UTI after primary unilateral pyeloplasty. Prophylactic antibiotics may be considered for the pediatric patients with risk factors above to prevent UTI.

## Figures and Tables

**Table 1:** Demographic and clinical characteristics of patients.

Characteristic	All (*n* = 504)
Age (month)	19.00 (5.35, 60.00)
Gender, *n* (%)	
Male	407 (80.75%)
Female	97 (19.25%)
Weight (kg)	11.50 (8.00, 19.70)
Height (cm)	83.00 (66.50, 112.50)
BMI	17.09 (15.59, 18.93)
Surgical modality, *n* (%)	
Open pyeloplasty	281 (55.75%)
Laparoscopic pyeloplasty	223 (44.25%)
Cr (*μ*mol/L)	26.00 (21.75, 34.50)
BUN (mmol/L)	4.08 (2.70, 5.10)
eGFR (ml/min/m^2^)	83.56 (73.24, 94.12)
Neutrophil (%)	29.30 (20.00, 41.45)
Lymphocyte (%)	59.40 (48.05, 69.70)
N/L	0.50 (0.29, 0.88)
APD (cm)	3.20 (2.60, 4.00)
Renal cortex thickness (mm)	2.00 (1.50, 3.00)
Caliectasis, yes/%	96 (19.05%)
Postoperative drainage, *n* (%)	
Internal drainage	355 (70.44%)
External drainage	149 (29.56%)

BMI: body mass index; Cr: creatinine; BUN: blood urea nitrogen; eGFR: estimated glomerular filtration rate; N/L: neutrophil/lymphocyte ratio; APD: renal pelvis anteroposterior diameter.

**Table 2:** Demographic and clinical characteristics of patients grouped by UTI and non-UTI.

Characteristic	UTI (*n* = 188)	Non-UTI (*n* = 316)	*Z*	*P*
Age (month)	6.72 (3.85, 17.50)	36.00 (9.50, 72.00)	-9.02	< 0.001
Gender, *n* (%)			2.38	0.017
Male	162 (86.17%)	245 (77.53%)		
Female	26 (13.83%)	71 (22.47%)		
Weight (kg)	9.00 (7.35, 11.53)	15.90 (10.00, 23.00)	-8.88	< 0.001
Height (cm)	70.00 (64.00, 84.00)	100.00 (72.00, 123.00)	-8.40	< 0.001
BMI	17.53 (16.00, 19.14)	16.76 (15.32, 18.63)	-2.70	0.007
Surgical modality, *n* (%)			2.38	0.018
Open pyeloplasty	92 (48.94%)	189 (59.81%)		
Laparoscopic pyeloplasty	96 (51.06%)	127 (40.19%)		
Cr (*μ*mol/L)	23.00 (20.30, 27.40)	29.40 (23.00, 38.00)	-7.54	< 0.001
BUN (mmol/L)	4.31 (3.30, 5.48)	3.02 (2.23, 4.51)	-6.96	< 0.001
eGFR (ml/min/m^2^)	82.50 (72.40, 92.03)	84.02 (73.89, 95.37)	-1.40	0.162
Neutrophil (%)	24.25 (18.00, 39.00)	33.80 (22.40, 42.70)	-4.26	< 0.001
Lymphocyte (%)	64.05 (51.00, 71.90)	56.80 (46.55, 67.45)	-4.07	< 0.001
N/L	0.38 (0.26, 0.77)	0.60 (0.34, 0.94)	-4.16	< 0.001
APD (cm)	3.20 (2.70, 4.15)	3.20 (2.50, 4.00)	-1.06	0.290
Renal cortex thickness (mm)	1.80 (1.28, 2.33)	2.20 (1.90, 3.40)	-6.50	< 0.001
Caliectasis, yes/%	44 (23.40%)	52 (16.46%)	1.92	0.055
Postoperative drainage, *n* (%)			6.33	< 0.001
Internal drainage	164 (87.23%)	191 (60.63%)		
External drainage	24 (12.77%)	124 (39.27%)		

BMI: body mass index; Cr: creatinine; BUN: blood urea nitrogen; eGFR: estimated glomerular filtration rate; N/L: neutrophil/lymphocyte ratio; APD: renal pelvis anteroposterior diameter. Statistical analysis was performed by the chi-square test or Mann–Whitney *U* test.

**Table 3:** Multivariate analysis of the incidence of postoperative UTI in pediatric UPJO patients.

Characteristics	*B*	S.E.	Wals	*P*	Exp (*B*)	95% CI	
Gender	-0.705	0.31	5.166	0.023	0.494	0.269	0.908
Age < 19 months	-0.032	0.013	6.118	0.013	0.968	0.944	0.993
Weight < 11.5 kg	0.137	0.055	6.292	0.012	1.147	1.031	1.277
Height < 83 cm	-0.06	0.022	7.302	0.007	0.941	0.901	0.984
BMI < 17.09	-0.164	0.069	5.737	0.017	0.848	0.741	0.971
Cr	0.031	0.022	2.057	0.152	1.032	0.989	1.077
BUN > 4.08 (mmol/L)	-0.285	0.088	10.437	0.001	0.752	0.632	0.894
Neutrophil (%)	0.03	0.021	1.98	0.159	1.03	0.988	1.074
Lymphocyte (%)	-0.018	0.023	0.606	0.436	0.982	0.938	1.028
Neutrophil/lymphocyte ratio	-0.267	0.239	1.248	0.264	0.766	0.479	1.223
Renal cortex thickness (mm)	-0.178	0.113	2.464	0.116	0.837	0.671	1.045
Surgical modality	0.142	0.245	0.336	0.562	1.152	0.713	1.861
Postoperative drainage	-1.978	0.303	42.751	0.001	0.138	0.076	0.25

BMI: body mass index; Cr: creatinine; BUN: blood urea nitrogen.

## Data Availability

The dataset used to support the findings of this study are available from the corresponding author upon request.
